# AI-DRIVEN Novel Approach for Liver Cancer Screening and Prediction Using Cascaded Fully Convolutional Neural Network

**DOI:** 10.1155/2022/4277436

**Published:** 2022-02-01

**Authors:** Piyush Kumar Shukla, Mohammed Zakariah, Wesam Atef Hatamleh, Hussam Tarazi, Basant Tiwari

**Affiliations:** ^1^Computer Science & Engineering Department, University Institute of Technology, Rajiv Gandhi Proudyogiki Vishwavidyalaya, Bhopal 462033, India; ^2^College of Computer and Information Sciences, King Saud University, P.O. Box 51178, Riyadh 11543, Saudi Arabia; ^3^Department of Computer Science, College of Computer and Information Sciences, King Saud University, P.O. Box 51178, Riyadh 11543, Saudi Arabia; ^4^Department of Computer Science and Informatics, School of Engineering and Computer Science, Oakland University, Rochester Hills MI USA 318 Meadow Brook rd, Rochester, MI 48309, USA; ^5^Department of Information Technology, Hawassa University, Institute of Technology, Hawassa, Ethiopia

## Abstract

In experimental analysis and computer-aided design sustain scheme, segmentation of cell liver and hepatic lesions by an automated method is a significant step for studying the biomarkers characteristics in experimental analysis and computer-aided design sustain scheme. Patient to patient, the change in lesion type is dependent on the size, imaging equipment (such as the setting dissimilarity approach), and timing of the lesion, all of which are different. With practical approaches, it is difficult to determine the stages of liver cancer based on the segmentation of lesion patterns. Based on the training accuracy rate, the present algorithm confronts a number of obstacles in some domains. The suggested work proposes a system for automatically detecting liver tumours and lesions in magnetic resonance imaging of the abdomen pictures by using 3D affine invariant and shape parameterization approaches, as well as the results of this study. This point-to-point parameterization addresses the frequent issues associated with concave surfaces by establishing a standard model level for the organ's surface throughout the modelling process. Initially, the geodesic active contour analysis approach is used to separate the liver area from the rest of the body. The proposal is as follows: It is possible to minimise the error rate during the training operations, which are carried out using Cascaded Fully Convolutional Neural Networks (CFCNs) using the input of the segmented tumour area. Liver segmentation may help to reduce the error rate during the training procedures. The stage analysis of the data sets, which are comprised of training and testing pictures, is used to get the findings and validate their validity. The accuracy attained by the Cascaded Fully Convolutional Neural Network (CFCN) for the liver tumour analysis is 94.21 percent, with a calculation time of less than 90 seconds per volume for the liver tumour analysis. The results of the trials show that the total accuracy rate of the training and testing procedure is 93.85 percent in the various volumes of 3DIRCAD datasets tested.

## 1. Introduction

### 1.1. Stages of Liver Cancer

In the biomarker selection of illness, the anatomical study of the liver and divisible lesions on magnetic resonance imaging are used in the selection of disease biomarkers. The diagnostic phases, succession initial and secondary hepatic tumours analysis are used [1]. The majority of initial tumours in different organs, such as the liver, colon area, and pancreatic region, commonly spread to the smaller structures in the organ. Consequently, frequent examination of the liver and its lesions is required in order to determine the main stage of a cancerous tumour. In addition to hepatocellular carcinoma illness, another major cause for infection of the liver area exists. In the liver area, this illness is referred to as a primary tumour disease, and it is one of the sixth most prevalent cancer diseases in the world, as well as the third most common cause of death for cancer patients globally [2–5]. Hepatocellular carcinoma is a kind of cancer that is genetic and molecular in nature, and it is most often caused by a chronically injured liver.

Various hepatocellular carcinoma illnesses have been identified and grouped into distinct groups based on their clinical presentation [6]. The progressive development of hepatocellular carcinoma is dependent on changes in tissue architecture and variations in vascular supply. Changes in the architecture of the tissue have been shown to accelerate the formation of additional tissue in the liver, which has been discovered via the use of medical imaging [3]. This procedure is dependent on the tumor cells' architectures and shapes, as well as their sizes. In clinical diagnosis, CT and MRI scans are utilised to examine liver cancer, with physical or semi-manual segmentation methods being employed in the process. These approaches are manual, highly operational, subjective, and time-consuming, and they need greater effort. Through the automated function, it is possible to decrease the amount of time spent on invention and radiologist improvement in computer-aided techniques, and to build unique segmentation methods. Automatic segmentation was performed on the combined liver and lesion area picture [7] to determine the extent of the lesion. The uneven segmentation in low contrast pictures between the liver and the lesion site has proven to be a significant hurdle for the researchers to overcome. When comparing hyper and hypo tumors, the contrast levels may be different, and the aberrant tissue development in the lesion may be different in different sizes and numbers of the lesion [8]. It is not possible to segment the liver area using the intensity-based technique because of the intricacy of the contrast variations seen across several testing instances. Cancer cells may have a variety of shapes, which reduces the efficacy of computational approaches that segment cancer cells. The suggested technique differentiates between cancer stages based on the structure of the tumor and the form of the lesion.

### 1.2. Shape Parameterization

In the image-based registration approach, the shape analysis is the most important component in segmenting the tumor area from the lesion region [4] and determining the location of the tumor. The memory of form, size, and tumor structure with respect to the metrics and landmarks of the liver cells is part of the image-based registration approach. Image-based registration technique This unique parameterization [9], which is based on the difference between the two objects, integrates the shape descriptor and the two-point inconsistencies in the picture in a single step. It has been shown that the prior approach for surface analysis may be used in a medical setting [5]. The parameterization of human organs is a difficult job to do throughout the segmentation phase. It is the sophisticated segmentation in medical imaging that is characterized by the parameterization of star-shaped objects in the abdominal region [10]. To lessen the deficiency impact, the suggested technique employs injective mapping in 2D surfaces, therefore removing the image's various areas [11]. The physicians, on behalf of the liver segmentation, validated the matching spots that would be used to include the statistical ship models throughout the training phase of the parameterization process.

### 1.3. Liver Segmentation

In recent years, researchers have devised a promising and new approach for detecting cancer and metastases. The most recent advancements in building and design have created new chances for metastasis to develop. Aside from that, dynamic bimolecular settings for various tumors are being researched. Types. Because of this, we may conclude that there is a causal relationship between gene expression levels in different tissues. It is possible to have a better understanding of how cancer develops early on biomolecular networks that have been connected to both normal and pathological processes by investigating various types of cancer. Cancerous states are a kind of cancer in and of itself. According to Ling et al. (2014), this hypothesis has been explored and he concludes that he has researched if there is a link between the mRNA terminologies of three distinct genes.

Following a random selection of the cancer-related genes PIK3C3, PIM3, and PTEN, the researchers discovered that the cancer had progressed. Since then, these coefficients have been tested in the area of cancer research. Diagnosis. While the patient was sick, the following observations were taken, and a decision was formed on how to treat him: A substantial correlation of 0.68 *r* 1.0 was found between the variables, indicating that the variables were related. PIM3 and PIK3C3 in breast cancer, PIM3 and PTEN in breast, kidney, and ovarian cancer, and PIM3 and PTEN in prostate cancer Malignancies of the liver and thyroid, as well as cancers of the breast and ovary, have been linked to PIK3C3 and PTEN mutations in the past. There is an assumption that the connections for early cancer detection are necessary in order to integrate the gene expression profiles of cancer networks to the clinical data that is already available. Biomarkers include things like cancer antigens and other such things. About ten to fifteen percent of all human malignancies are caused by cancers. Viruses are also responsible for certain cancers. A technique known as massively parallel sequencing has been found to be successful in both malignancies and normal tissue for the discovery of new viruses and the interactions between them.

### 1.4. Analyses of Hepatic Tumors (1.4)

According to MICCAI, the problem of differentiation was first raised in 2008, at a time period that included the segmentation of liver tumors [12, 13]. It researches and develops different disease segmentation strategies as well as contrast improvement approaches for tumor segmentation from healthy hepatic parenchyma utilizing computed tomography images. Contained Participants were given an introduction to data and measuring procedures. Tumor segmentations were tested using five semi-automated and four automatic methods. The approaches for the liver differentiation competition were estimated using equivalent metrics. To separate tumors [14], Standard Graph Cutting techniques and the watershed algorithm were utilised suitably, much as they did for liver segmentation methods, to provide the most accurate measuring tool. A similar number of semi-automatic approaches are used; the most frequent are adaptive thresholds and morphologies, voxel identification and dissemination, and pixel identification, among others. In order to segment tumors, neural network technology and an ad boost taught community discriminating by artificial intelligence and picture recognition are the most effective approaches [15].

### 1.5. Our Approach

We will apply new automated technologies for the segmented liver, which will continuously improve contrast and imaging artefact removal while reducing the amount of time required. The resilient parameter of 3-D surfaces is presented for use in the segmentation procedure among abdominal organ pictures in order to increase the contrast between the two images. On the surface of objects, the 3-dimensional plane is represented in the form of the *x*, y, and *z*-axis when a closed planar curve is drawn on the surface. This representation of the space eliminates the frequent issues associated with the surface parameterization of concave objects. In order to eliminate noise type descriptors throughout the segmentation process, we use rotational and resilient approaches. A shape-driven geodesic active contour is used to improve liver segmentation after the first segmentation has been identified [16]. It is necessary to detect and treat hepatic tumours at an early stage in order to reduce the risk of mortality in a given individual. The features of tumour candidates are retrieved, and the support vector machine Algorithm is used to classify the candidates. It has been determined that the suggested segmentation approach outperforms and can be compared to current algorithms on a number of datasets with varying age limitations. In the case of hepatic tumour imaging, the segmentation of the liver and the computation of tumour measurement are difficult. Patients with abnormal livers may be traced down and identified using the automated liver cancer analysis method, even if their photos have poor image quality or are incorrectly labelled.

Because of the limited amount of medical image data that is currently accessible, as well as the limits imposed by GPUs, the exploitation of 3D data may result in overfitting challenges in certain cases. This research proposes an enhanced VNet and a 2.5-dimensional convolutional neural network VNet WGAN to acquire context information from 3D data in order to achieve end-to-end segmentation of liver images. The enhanced VNet and the 2.5-dimensional convolutional neural network VNet WGAN are used to achieve end-to-end segmentation of liver images. Among their key tasks are the following:

In this step, two convolution kernels are used in series with the input being the stack of slices and their upper and lower adjacent slices, and the output being the segmentation map corresponding to the central slice to fully extract the intralayer and interlayer information that will be used in the 3D liver model.

1. The input being the stack of slices and their upper and lower adjacent slices, and the output being the segmentation map corresponding to the central slice Despite the fact that segmentation accuracy remains high, geographic considerations may be able to assist reduce the amount of memory used and the amount of computation required.
2. In order to make full use of the network's high-level and low-level characteristics, a chain residual pooling module is added to the VNet network's long-skip link structure in order to maximise the use of both high-level and low-level features. This enables for the accumulation of more detailed semantic information as well as an increase in the accuracy of liver segmentation by a large margin.
3. Incorporate the boundary loss function into the basic WGAN generator network to make up for the lack of attention paid to the marginal pixel accuracy of the Dice loss function in the preceding step by including the boundary loss function. By including the composite loss function of boundary and Dice weighted fusion into the equation, the segmentation ability of the model is enhanced from the region and the boundary, respectively.

The ability to take random inputs and generate the appropriate output, as well as execute efficient inference and learning processes, is shown by fully convolutional networks that are cascaded. Adversity is a part of life. Through the use of this approach, the function is evaluated over the whole image frame. Patch-based approaches, as well as segmentation objects, are also utilised in this application. Instead of processing patches, the network processes entire pictures, reducing the amount of time spent on the network and the requirement to choose fertile areas in order to minimise the amount of repetitive reproduction estimate when patches overlap, resulting in an increase in the size of the final picture. The House of Representatives passed a resolution. Furthermore, many scales are integrated by connecting them together in ways that combine the most recent detection with lower layers with higher resolution. These measurements are made possible by combining numerous scales. This kind of fusion may be created in a number of shapes and sizes. This procedure generates a heat map of the lesion, which may then be used to diagnose it if necessary.

The following are some of the significant contributions made by this paper:

- It is our intention to offer the Cascaded Fully Convolutional Neural Network, which will be utilised for the detection and segmentation of liver cancer.
- It is being developed with the assistance of a deep learning system that is effective in segmentation and classification. Tumors of the liver are categorised based on where they are found on the body.
- The experimental results reveal that the proposed HFCNN is successful in that it makes use of the dataset to achieve high overall performance.

It is also anticipated that the suggested approach would assist the individual with the pace at which tumour cells develop, which will aid in the early identification and diagnosis of cancer. The following sections are included in the paper that was submitted.  Section 2 contains a list of comparable works that are discussed in the context of the background study, and Section 3 contains the methodology for the proposed work.  Section 4 discusses the experimental examination, and Section 5 summarises the findings and discusses future research opportunities.

## 2. Related Works

In CT imaging of the liver and liver lesions, there are numerous techniques for segmenting the organ that have been developed in both interactive and automated approaches. [17] Two benchmarks were conducted on liver and liver lesions segmentation at the MICCAI 2007 and 2008 Sessions, which were both published in [18]. The statistical model forms were the focus of the concerns discussed throughout the workshop. In addition, the workshop focused on grey levels and lesions texture analysis [18], which were also discussed. Otsu segmentation is a method that has lately become popular for graph cutting and level setting in pictures of liver cancer. However, because of the rise in velocity and intensity level, as well as the poor contrast in CT data, these approaches are not routinely employed in clinical settings. Interactive approaches are continuously being developed to address these flaws and strengthen their defences against future attacks. Target identification, classification, and segmentation are among the computer-vision problems that the academic community is becoming increasingly concerned with, thanks to algorithms such as cutting-edge techniques, Deep Convolutional Neural Networks (CNN) [19], which are used to do these tasks. Above all, CNN techniques have been shown to be the most user-friendly and most novel methodology for the segmentation of liver cancer in CT images as well as the segmentation of lesions in CT images, and they are now the most widely used.

According to Rong Zhu et al. [20], an image processing filter application of an improved anisotropic diffusion was developed, showing that anisotropic diffusion filters are the most frequent strategy for noise reduction. This study describes a more efficient approach for the anisotropic diffusion filter, which may be used to remove salt and pepper noise from photos. Ravi S, et al. [21] developed Morphological Operations for Image Processing, Understanding, and Applications, which they put into practise. The purpose is to remove any defects that may exist within the picture structures. Wassim Abdulrahman and colleagues [22] The term “Segmentation of Liver Tumors Using Image Processing” refers to the process of distinguishing specific parts of the liver in abdominal CT scans. When it comes to retrieving the tumor's location from CT scans, a new method has been developed. Amit Verma and colleagues, [23] “Techniques for Detecting Tumors Using Digital Imagery The background analysis in the segmentation of tumour cells is provided by the survey.” If you compare the performance of this method to other existing methodologies, it is the most effective at finding and categorising cancers. According to Jinshan Tang et al. [24], an Adjustable Anisotropic Noise Reduction filter in MR images was developed, and it was recommended that an adaptive threshold range be used in the stepped-forward anisotropic diffusion filter. A transparent diffusion with an anisotropic probability-pushed memory system is proposed to tackle the over filtering problem by selecting a tissue and an overall metaphysical impact from a large number of possible options. The proposed technique has been tested in real MR pictures, and the results have been outstanding.

Alireza is an anisotropic diffusion filter that is used to cancel noise in the input picture throughout the processing steps. R. Lin and E. K. Wong [25] developed “Morphological operations on quadrants represented by images,” which included a series of guidelines for performing direct morphological operations on quadrates represented by images as well as creating dilated and eroded snap images representing quadrants that were based on quadrates. Ruchika Chandel et al. [26] defined the segmentation algorithms and technique used for illustration of filter in embodiments and smoothing, as well as the smoothing algorithms and technique “Image Filtering Algorithms and Techniques Image smoothing, also known as image smoothing algorithms and techniques, is one of the most significant image dispensation techniques that is widely used. According to N. Howard and colleagues [27],” “a novel completely automated liver and tumour fragmentation system with a morphological operation” was developed for a numerical hepatocellular carcinoma detection method that was both high-sensitive and low-specific in its imaging. The present system came to the conclusion that segmentation using 2-dimensional photos is less accurate and requires more time to analyse than 3-dimensional images.

Prior to anything else, it's important to segment the liver so that the tumour on the CT image may be appropriately segmented. The segmentation of a tumour, and much more so the segmentation of a tumour in combination with the liver, is substantially more complex than it seems at first glance. General practitioners (GPs) will have a tough time visually distinguishing the liver and tumour from other undesired cells and nearby organs if they do not have specific training in this area. When a CT picture has low contrast, a dynamic size, non-uniform intensity, and an assortment of artefacts, segmenting the liver and tumour is considerably more challenging, even for an experienced radiologist or doctor. However, despite the fact that segmentation conducted by professionals is accurate, it requires a large investment of time and effort. Apart from that, specialists in liver cancer who are capable of executing exact and fine segmentation are rare to find, and they are especially inaccessible to the people of impoverished countries, where the issue of liver cancer is more frequent. A more exact and effective algorithm for tumour segmentation, as well as algorithms for assessing tumour size, shape, and location, are required as a result of the presence of these problems. A range of semi-automatic and manual procedures have been developed in order to segment the tumour in the liver and determine its location. Given that each of these systems is dependent on human interaction, they are all susceptible to user error, individual bias in feature selection, and time lag. A totally automated segmentation technique, capable of segmenting both the liver and the tumour in a single run, is necessary in order to do this. In this way, a doctor or radiologist may reduce reading time, increase detection sensitivity, enhance diagnostic accuracy, and discover malignancies early in the process without interfering with the patient's health. Following extensive testing, these technologies may also be used in instances where there is a paucity of competence in liver imaging. In recent years, researchers have concentrated their efforts on creating a wholly automated system that can generate accurate and timely forecasts of liver tumours while saving a large amount of time and effort on the part of the researcher. The benefit of entirely automated approaches is that they evolve over time as a consequence of their output as well as the absorption of diverse conditions and inputs into the system as the system matures. A large number of research that have lately been published provide credence to this notion.

When using 3-dimensional pictures with the geodesic active contour approach, the suggested methodology boosts the accuracy rate while simultaneously decreasing the segmentation processing time, hence eliminating these flaws.

## 3. Methods and Materials

### 3.1. Overview of Our Proposed Segmentation Processing

380 patients contributed a total of 2012 CT images, which was collected from 398 individuals. Three hundred and thirty-three patients with Hepatocellular Carcinoma in Adults were found, resulting in a total of 591 CT pictures; three hundred and twenty-five patients with Hepatocellular Carcinoma in Children were identified, generating a total of 1421 CT images In order to establish the final diagnosis of these photographs, and in the absence of surgical intervention, the results of the lesions were utilised to establish the facts, so enabling the data to be regarded as reliable. A qualified physician additionally changed the window width and window level of the CT scans shown above to guarantee that the cancer tissue could be clearly seen in each image. Using these modifications, the cancer tissue was clearly seen in each image. The Digital Imaging and Communications in Medicine (DICOM) data was utilised to construct the final picture after it had been normalised to a grayscale image with a grayscale value of 0–255 according to the appropriate window width and window level. GIF files include the jpg extension, which stands for grayscale picture format. Using a medical professional's hands, the shape of the liver region was created in the CT image. The intended work will be divided into three main phases. The first stage is concerned with the preprocessing and segmentation of data. The graph cut approach is used in the second phase to gather features based on the segmented area of lesions that have been identified. In the final third stage, two cascaded fully convolutional neural networks with Training and Testing pictures are used to solve the problem.

In Figure 1, we can see the suggested workflow, which is made up of all of the various processing units. For the purpose of performing early-stage detection of liver cancer, the training and testing stages are carried out.

### 3.2. Shape Analysis and Surface Parameterization

As a S shape function, a 3D equivalent of a curve characteristic was utilised to equate closed planar curves in order to discover structural discrepancies in the data. S is the cross section area of the interior of the turn and “seed” at the given point *p* on a planar curve, in further detail (a sphere centred at p). If the instantaneous parameterization of the two curves is adequate, a S curve C may be used for both regional and global comparisons of the two curves, assuming that the two curves are sufficiently parameterized (at any corresponding position on two matched curves). Var is the volume of the C-intersection, and the Radius *r* radius seed sphere matches the size of the C-intersection. The influx of digital goods served as a consoling element in the situation. The mode descriptor is invariant with respect to architecture and resilient to noise.

Our method makes point-to-point comparisons across numerous surfaces by using the organisation of an entire class of substances, as seen in Figure 2, which we refer to as planar-convex arrangement. We think that livers are included in this category. An aircraft P to O is defined as a planar-convex object O in Rn that is defined as a stop up the surface when a set of equivalent hyperplanes P is present, allowing us to acquire an unique closed planar curve in any cross section of an aircraft P to O. This is how we refer to any collection of hyperplanes that are parallel to the O as “convexity planes.” We balance two things by coordinating their principle components, and we orient a collection of symmetrical points to the vertices of a square centred on the object's greatest primary constituent by coordinating their principal components. Using this method, we may locate numerous sets of the identical plane, which intersect the object with normals that span throughout a hemisphere equally; we sampled a dodecahedron with 32 vertices to demonstrate the concept. Afterwards, we determine whether main plane (*x*, *y*, or *z*-plane) is more successful in mapping the parallel planes, as indicated by equations (1) and (2);

(1) $$\begin{array}{c} S\left(p\right)=\frac{\int_{C}^{1}xV_{r}\left(p,x\right)\text{d}x}{\int_{C}^{1}xV_{r}\left(p,x\right)\text{d}x}. \end{array}$$

Each plane's link to the liver, as well as the regular number of associated workings, are next thoroughly analysed. This approach will identify the smallest possible sum of average mechanisms in the axis/plane of the two compounds. As a result, the location of matching convexity planes P between two identical objects (as previously specified)—liver segmentation and testing from CT scans of sick patients, and cancer from CT scans of the same patients—can be established. [28] The surface of each convexity plane is sampled using a user-defined number of divisions, and the points of these partitions are projected onto the surface of the goal, with each partition representing a point on the surface of the target. During the demonstration, you will be shown an example of liver parameters. When comparing two items or lives, these assessments, also known as “parameterization points,” are made in relation to one other. In order to study the outcomes, we compute the form function S at each parameterization point and transfer its value onto the surfaces of each entity so that the consequences may be seen. When S is generated from the coordinated preparation surface, it is averaged at both ends, and it is normalised between zero and one on the scale of 0 to one. Using the most elementary parametrization, this is seen in Figure 3.

### 3.3. Segmentation of Liver Tumors and Lesions

The first liver segmentation reveals regions on the surface of the liver that have an uncertain structure based on the surface points that were matched to the training results in the first step. S has a cutoff of 0.5, and component analysis is used to give unique marks to each uncertain location, allowing for any degree of intra-patient variability to be accommodated in the study. Because the livers were largely segmented by the original approach, the seeds were placed in the centre of the label, and a rapid marking level was used to “crease” the segmentation based on the sigmoid of the CT images [29], the seeds were placed in the centre of the label. A geodesic contour with dynamic geometry refines the segmentation. The technique is repeated until the volume changes by S 0.5 or until the volume changes between iterations. To characterise timid hepatic masses, a graph-cut method segmenting the liver is utilised, as recommended by the process, to segment the liver. In their simplest version, the graph cuts are affected by the shrinking bias issue, which is especially problematic for the segmentation of enlarged and tiny structures such as blood arteries and some tumour shapes. Tumors and veins are quite diverse from case to case, and the segmentation of abdominal organs with formations has improved as a result of the diagram cuts. Tumors, on the other hand, are often elliptical and curved [30]. It is necessary to compute the tumour vessels and blobs using equations (2) and (3).

(2) $$\begin{array}{c} E_{\text{vessels}}=-\ln\ln\underset{\sigma }{\max}\left(\sigma^{2}v\left(p,\sigma \right)\right),\;\\ \text{with }v=\left\{\left|\lambda_{2}\right|\right.+\lambda_{1},\text{ if }\lambda_{1}<0\;\left|\lambda_{2}\right|-\frac{\lambda_{1}}{4},\\ \text{if }\lambda_{2}<0<\lambda_{1}<4\left|\lambda_{2}\right|. \end{array}$$

(3) $$\begin{array}{c} E_{\text{blobs}}=-\ln\underset{\sigma }{\max}\left(w\right),\\ \mathrm{with}\;\lambda_{3}>0;\\ w=e^{-\left(\lambda /\lambda 3^{-1}\right)}. \end{array}$$

We have reduced the size of the picture by segmenting it using limits for increased vasculature, tumour opacity, and Hessian shape. This allows us to emphasise tiny elongated veins and circular tumours on several scales using our segmented image. The Hessian's values (*p*1 > *p*2 > *p*3) at point *p* highlight major type restrictions that may be used to enhance vascular segmentation and lower the number of false-positive tumours detected. In the graph description, the following force conditions are utilised to describe the graph. Improved hepatic arteries were removed before to tumour segmentation in order to reduce the number of false-positive tumour detections. By standardising the overall volume of the liver, the aggregate quantity of tumours was computed for each patient in order to measure the pressure exerted by tumours and follow the progression of metastatic hepatic cancer [31].

### 3.4. Correction of Liver Segmentation

We have reduced the size of the picture by segmenting it using limits for increased vasculature, tumour opacity, and Hessian shape. This allows us to emphasise tiny elongated veins and circular tumours on several scales using our segmented image. The Hessian' values (*p*1 > *p*2 > *p*3) at point *p* highlight major type restrictions that may be used to enhance vascular segmentation and lower the number of false-positive tumours detected. In the graph description, the following force conditions are utilised to describe the graph. Improved hepatic arteries were removed before to tumour segmentation in order to reduce the number of false-positive tumour detections. By standardising the overall volume of the liver, the aggregate quantity of tumours was computed for each patient in order to measure the pressure exerted by tumours and follow the progression of metastatic hepatic cancer [31].

(4) $$\begin{array}{c} E\left(A\right)=E_{\mathrm{data}\;}\left(A\right)+E_{\mathrm{enhance}\;}\left(A\right)+E_{\mathrm{shape}\;}\left(A\right)+E_{\mathrm{boundary}\;}\left(A\;\right), \end{array}$$

(5) $$\begin{array}{c} E_{\text{data }}\left(A\right)=-\sum_{p\in O}^{x}x\;\ln\left(\frac{\sqrt{P\left(I_{p}|O\right)}}{\sqrt{P\left(I_{p}|O\right)}+\sqrt{P\left(I_{p}|B\right)}}\right)-\sum_{p\in B}^{b}P\;\ln\left(\frac{\sqrt{P\left(I_{p}|B\right)}}{\sqrt{P\left(I_{p}|O\right)}+\sqrt{P\left(I_{p}|B\right)}}\right), \end{array}$$

Also included in equation (4) through equation (6) are the voxel intensity and probability of artefacts, as well as the surrounding field, Euclidean distance, and the normal fluctuations in image noise, among others. New language in this formulation refers to the local notion that punishes voxels that do not adhere to the dissimilarity in sharing of better tumours with stable liver parenchyma models, as defined by training. Our index encourages darkish spots within the liver to be identified as tumours since the liver is a better option than cancer in terms of survival. During training on different liver cancers, the relationship between the healthy (background) liver and the diseased (object) liver alters as a result of the training.

(6) $$\begin{array}{c} E_{\mathrm{enhance}}\left(A\right)=\sum_{\left\{p,q\right\}\in N_{p}}^{q}x\frac{1}{1+{\left({\left(I_{\delta }^{\prime }-I_{i}^{*}\right)}^{2}/2\sigma^{2}\right)}^{2}} \end{array}$$

where the value of the intensity is specified, and the value of the intensity at the context is specified, the intensity (B). We believe that the surgery is not intended to segment the hepatic vasculature since the improvement is unusual in our circumstances. The traditional geodesic active contour model was utilised to simulate the minor segmentation of tumours in order to maximise their segmentation using a speed spread parameter of five and a curvature parameter of two and a half. By normalising the overall volume of the liver, the total volume of tumours was estimated for each patient in order to measure the pressure exerted by tumours and follow the progression of metastatic hepatic cancer. The absolute difference between the tumour burdens estimated manually and those computed automatically is used to calculate the tumour burden error. The effects of artificial Gaussian noise and body rotation on an axial flat surface were reported and compared with ground reality in order to investigate the reproducibility of estimating tumour burden under the influence of image noise and patient location variations in order to research the reproducibility of estimating tumour burden. When it comes to accentuating circular, multi-scale tumours, the Hessian type is required. Hessian' principles provide certain form limitations that may be used to enhance tumour division while simultaneously reducing the number of false positive tumours. Eqn. 7 has the following energy terms, which are shown graphically in the diagram.

(7) $$\begin{array}{c} E_{\mathrm{shape}}=-\ln\underset{\sigma }{\max}\left(w\right). \end{array}$$

We believe that the surgery is not intended to segment the hepatic vasculature since the improvement is unusual in our circumstances. The traditional geodesic active contour was utilised to simulate the minor segmentation of tumours in order to maximise their segmentation with a pace propagation parameter of five and a curve parameter of two and five, respectively. When the entire liver volume was normalised, the total volume of tumours was computed for each patient in order to measure tumour pressure and follow the progression of metastatic hepatic cancer. For the tumour burden error, the absolute difference between the manually computed tumour load and the automatically calculated tumour load is calculated. On the axial level surface, the fake Gaussian cacophony and body rotations were recorded and compared with the ground reality in order to investigate the repeatability of assessing tumour load in the presence of picture noise and patient location alterations.

### 3.5. Tumor Features and Classification

A set of 157 characteristics is automatically analysed for individual tumor applicants to classify detections. This involves the scale, development, 3D forms, and 3-D texture as seen in Table 1.

The collection of functions in Table 1 was too old to preserve the ideal combination of components to separate accurate positive detections from false-positive detections (TP) because of the large number of classification characteristics that were employed (FP). Due to the fact that various skin textures might overlap and connect together, the classifier must identify the most insightful and distinct characteristics. We can pollute or impair the specific details found in these features if we quantify correlations between exercise samples, which may result in low classification precision. If we quantify correlations between exercise samples, which may result in low classification precision, we can pollute or impair the specific details found in these features. We have conducted tests with a collection of functions, using the methods of least redundancy and maximum application, in this regard (mRMR). mRMR is a feature selection tool that is state-of-the-art in the field of biomedical data processing. Selecting features based on common knowledge and reducing duplication between attributes according to the maximal statistical dependency criterion are two of the benefits of using this method.

### 3.6. From AlexNet to U-Net

Using a totally convolutional network design for semantic segmentation, Long et al. [32] developed the first such architecture. To create dense predictions by pixels, the researchers use a fully coevolutionary layer structure to replace the last wholly linked layers of a classification network, such as AlexNet, with entirely coevolutionary layers. For the final entirely coevolutionary layers to be adjusted in order to accommodate the input measurements, The AlexFCN (Fully Convolutional Network) improves upon the prior work by allowing full-size medical slices to be projected pixel-wise rather than patch-wise. Using 3D CAD data sets, the AlexFCN training curves (without combining classes) were created. The convergence of all training curves to a stable state occurred quickly when the training and assessment overlapped. AlexFCN has a considerable excess of class equilibrium in both training curves, with Dice overlaps in liver examination exercise knowledge of 90 percent and accidents of 60 percent, respectively, in AlexFCN.

When it comes to examination occasions, the lesion Dice of 24 percent is equivalent to a bad result. It asserted that the class balance was not required in order to resolve their problem with natural picture segmentation. Using AlexNet weights trained on actual photos, for example, might explain why the model was utilised pre-trained in the first place. For training and testing photos, data from ImageNet is utilised. Many medical applications, however, need the employment of class balancing because pre-trained networks of real pictures are insufficiently utilised and because the class of attention is less often included in the dataset than the other classes. Preparation and monitoring of Dice for the liver and lesions both improved modestly, with 78 percent of the liver and 38 percent of the lesions being successfully completed on the first attempt. Additionally, the U-Net has a better pattern of skipping connections across different stages in the neuro-network, in addition to its 19-layer breadth. During the present phase of activations, spatial awareness is accessible in the early stages of the neural network. Spatial information is passed to semantic information at subsequent levels via the neural network, at the price of specific knowledge of the placement of certain structures. Using the original U-Net design, for example, a 388 × 388 input picture that would otherwise be a bottleneck is reduced to a 28 × 28 output image. As subsequent stages will merge geographic data from above with neural networks, skip-links will be used to assure later point utilisation and transfer of spatial and semantic data. In later phases, the neural network may make use of semantics and spatial sequencing to make deductions.

### 3.7. Changes from Fully Convolutional Network to Cascaded Fully Convolutional Network

In the soft mark probability maps P, we have been using the U-Net architecture as a framework. The U-Net design allows for accurate pixel estimation by combining spatial and temporal data into a 19-layer co-evolutionary network architecture—the training U-Net curves in the 3D CAD data set—and merging the results into a single network architecture. In addition, the cumulative lesion segmentation effectiveness has been increased to 53 percent, according to Research Dice. The U-Net has mastered the ability to distinguish between liver and lesion at the same time. One of our most significant innovations is the cascade training of FCN to learn unique features just once during training in order to complete a segmentation assignment, which results in improved segmentation efficiency overall. The approach was developed as a result of the fact that U-Nets and other forms of CNNs recognised the hierarchical structure of the input data. Instead of planning human-crafted face appearances for the separation of distinct tissue kinds, the neural network' stacks of layers are adjusted towards the chosen categorisation in a data-driven manner, rather than by hand. By cascading two U-Nets, U-Net learns from a general CT abdominal scan filtering that is specific to the identification and segmentation of the liver, rather than from a general CT abdominal scan filtering. Figure 2 shows U-Net putting together a filtering process to identify lesions from the liver at the same time as the previous figure. Additionally, the ROI of the liver contributes to the eradication of lesions. We're teaching one network in the abdominal area of the liver, specifically (step 1). It is the only emphasis of this network's research to identify and investigate discriminating traits in liver-background segmentation. After that, we train a second network to segment the lesions in the liver image that we have obtained (step 2). After being segmented in Step 1, the liver is cropped and re-sampled in Step 2 in order to get an input dimension that is suitable for the cascade U-Net. It is possible that the second U-Net will concentrate on learning discriminating properties of the lesion rather than on segmenting the liver history.

  Initialize the segmentation process
  Begin with features of segmentation image
  Let *x* be feature of the pixels
 
*y*_*k*_=*g*_*m*_(*y*_*m*−1_)*be the neuron layers*
 
*While x feature >y*_*k*_
 
*y*_*k*_=Re*LU*(*x*_*m*_ ⊗ *y*_*m*−1_+*C*_*m*_)
  then
 
*f*(*y*)=*m*^*y*^(0, *y*)
  End

where *y*_*m*_ represents a series of convolution operations for each layer. *y*_*k*_ represents the output of layer *m*· where *x*_*m*_ is the convolution kernel weight, *c*_*m*_ is the offset value, and ⊗ is the convolution operation.

### 3.8. Effect of Class Balancing

One of the most important steps in FCN training is to balance the needed classes with the class in the data following the pixel frequency of the target. In contrast to [33], we discovered that preparing the system to segment microscopic structures such as lesions is not practicable without class complementary, owing to the substantial class inequity, which is typically in the range of 1% for lesion pixels, and hence not feasible without class complementary. As a result, we have included an additional weighting element in the cross-entropy loss function *L* of the FCN.

(8) $$\begin{array}{c} L=-\frac{1}{n}\sum_{i=1}^{N}n\omega_{i}^{\text{class}}\left[{\hat{P}}_{i}\log\;P_{i}+\left(1-{\hat{P}}_{i}\right)\log\left(1-P_{i}\right)\right]. \end{array}$$

*Pi* denotes the likelihood of voxel *i* belonging to the center, ${\hat{P}}_{i}$ represent the position truth. We chose *class i* to be PP*i* 1*i*-${\hat{P}}_{i}{\hat{P}}_{i}$ if ${\hat{P}}_{i}$ = 1 (see Figure 4).

## 4. Experimental Results

We found that the initial segmentation approach was less successful than previously reported [34] because of tumours and other items in our data, as well as the conflicting retrieval of contrast-enhanced pictures. The use of liver-to-liver parameterization in conjunction with active geodesic contour considerably decreased the fraction of volume mistakes in both situations of severe fragmentation failures and those needing modest changes. An example of segmentation from an artifact-free event, a somewhat erroneous segmentation, and a substantial segmentation malfunction are all shown in Figure 5, along with their corresponding type photos and performance during the final repair. With our methods, we were able to enhance the segmentation of crucial instances with tumours while also minimising mistakes in well-secreted livers by a large margin. Since the first and previous segmentation, there has been no arithmetical difference in the segmentation of the liver since the first and prior segmentation.

When manual segmentations were performed on the 14 instances, the usual liver tumour strain was found in 6.6 percent to 9.0 percent and 7.1 percent of the cases when automated segmentations were performed. According to the Wilcoxon rank-sum test, there was no statistically significant difference between the measurements.  Figure 6 depicts the change in liver and tumour volume over time, as well as the tumour load, which is significant for many patients.

When we used 3D CRF to our segmentation issue, we were able to demonstrate statistically significant increases in the quality of the segmentation. Because of this, tuning hyperparameters such as 3D CRF requires a significant amount of effort and time. With unintentional search, it is difficult to locate a hyperparameter set that is generalizable to concealed possessions with diverse structure in figure and exterior, such as an HCC lesion. The 3D CRF has also been successfully completed for the treatment of diverse brain lesions. The introduction of new CRF hyperparameter learning into the training phase was a complete success. When this method is combined with additional words that include prior knowledge of the problem, the CRF's performance for that job may be enhanced.

A Cascaded Fully Convolutional Neural Network for liver tumour detection and segmentation has been proposed for the first time, and it is expected to be widely used in the future. In the system, there is a training phase as well as a testing step for each neural network that is included. The use of data augmentation techniques throughout the training phase helped to increase the overall quality of the CT data that was gathered. It is next necessary to feed the expanded information into the neural network system in order to acquire a qualified framework. This process is known as input data feeding. Our feature extraction strategy comprised the testing of a range of CNN layers in an effort to develop a more effective feature extraction network, which was ultimately successful. This research seeks to overcome the limitations of present spatial 3d information in the identification of neural networks, which are not fully explored at the time of publication. Throughout the Proposal phase, the ideas for the field have been generated from a pyramid structure in order to capture lesions of varied sizes.

The approach is referred to as return on investment (ROI). In contrast, it has been established at this level that a texture classifier can be utilised to distinguish between normal and pathological liver lesions in ROIs collected during the study. Hepatocellular carcinoma (HCC), liver cysts, and hemangiomas irregular hepatic lesions have been distinguished using abstract functions at the classification detection stage, as well as at the classification detection stage and the classification detection stage, respectively. The training phase of this project included a number of iterations that were carried out in order to get a more accurate model structure. During the testing stage, the system was eventually assessed based on the data collected from another batch of CT imaging.

It is obvious from Table 2 that the various segmentation strategies have a variable accuracy rate in terms of classification. Transfer learning using neural network models that have already been trained is a frequent idea in deep learning. When training on a new job, such as medical volume segmentation, neural networks [8] trained on previous tasks, such as a data set for natural image classification, may be used as a starting point for weights of the network to be trained on. The underlying premise of these discoveries is that the initial layers of neural networking for many tasks or datasets uncover a comparable notion to observe crucial systems such as blobs and verges, based on the same theory. When pre-trained models are used, these ideas are not taught from the beginning from scratch. We employ pre-trained U-Net models that have been trained on cell segmentation data to assist our researchers on creating their preparation [7] for our studies, which includes an erudite liver and lesion concept. We have made our taught model on liver and damage segmentation available for download [6].

According to the different current algorithms, as seen in Figure 7, the proposed Unet architecture has the highest rate of accuracy (94.025 percent), as well as the lowest rates of sensitivity and specificity (both 0.5 percent). Due to the longer calculation time required by the other current method, the accuracy rate of the system is diminished.

According to Figure 8, when it came to identifying liver cancer, the sensitivity and specificity were 94.4 and 77.8%, respectively, when compared to other tests. Using an AUC of 0.8070 and a threshold value of 28.35, the sensitivity and specificity for the diagnosis of liver cancer were 83.3 percent and 77.8%, respectively, showing that the test was both highly sensitive and specific for the disease.

According to the classification stages, the habitats of the people have the most influence on the development of liver cancer. The prediction rate of a person in their everyday life is shown in Figure 9 with regard to their age and environment, respectively. Alcoholism increases a person's risk of developing liver cancer, which is particularly dangerous for men. This diagnostic tool may be able to detect liver cancer in its early stages, which would aid in the decrease of the fatality rate.

## 5. Conclusion

Cascade FCNs and 3D CRFs are trained for automated CT volume placement and to co-ordinate the volumetric secretion of illness and injury in order to get optimal results. It is cutting-edge technology that we are proposing to use. We are making our qualifying models available under open-source permission in order to further medical applications in CT data 8. Furthermore, we built and evaluated dense 3D CRF as post-processing measures to inspect a deep medical picture based on learning in order to investigate a deep medical image based on learning. Furthermore, our suggested technique, which involves cascading numerous FCN, has the potential to be applied to many organ segments. The use of additional waterfall FCNs as prospective work ROI for lesions in order to identify the malignancy of the lesions and to do advanced operations. An increase in the use of unfavourable networks may help to enhance the accuracy of segmentation. It is possible to separate the heterogeneous quantities of CT and DW-MRI from different scanners and the specified methods into smaller groups of under 100 apiece. Let us bring this to a close. For automated liver analyses and associated lesions, CFCNs are promising approaches in clinical practise. They are also being studied extensively in medical research [32, 35–42].

## Figures and Tables

**Figure 1:** Proposed workflow.

**Figure 2:** An example of the form descriptor on 2-D closed curves. The seed is a circle that intersects the objects (here a square and a wider circle) (here a square and a larger circle). Provided a suitable parameterization of the two closed curves, their point-to-point local discrepancy can be measured.

**Figure 3:** Parameterization points are highlighted as small cubes on the surface of a liver with an irregular shape. These points allow point-to-point correspondence between two shapes.

**Figure 4:** Multiview fusion of proposed cascaded network.

**Figure 5:** Segmentation of trained and tested features.

**Figure 6:** Cascaded Convolutional Neural Network of trained and tested features.

**Figure 7:** Prediction rate of trained and classified tumor cells.

**Figure 8:** ROC of enhanced UNet architecture with geodesic active contour.

**Figure 9:** Classifier stages with respect to routine habitat.

**Table 1:** Automated tumor features.

3D feature	Descriptor	Explanation
Tumor volume	Size	Volumetric size
Tumor diameter	Size	Linear size
Tumor size ratio	Shape	
Tumor binay elongation	Shape	Rato of the size of bounding box and real size
Tumor intensity	Shape	Enhancement of tumor region
Edge intensity	Enhancement	Enhancement of healthy region
Cluster	Enhancement	Skewness
Prominence	Texture	Skewness
Edge cluster shade	Texture	Skewness
Correlation	Texture	Complexity
Energy	Texture	Complexity
Entropy	Texture	Roundness
Tumor blobness measure	Texture	Heterogeneity
Inertia	Texture	Heterogeneity
Edge inertia	Texture	Heterogeneity
Tumor inverse difference	Texture	Heterogeneity
Edge inverse difference	Texture	Heterogeneity

**Table 2:** Segmented Tumor Parameters using Cascaded Convolutional Neural Network.

Approach	VOE	RVD	ASD	MSD	DICE
	%	%	%	Mm	%
UNET	39.27	87	19.4	119	72.9
Cascaded UNET	12.8	−3.3	2.3	46.7	93.1
Cascaded UNET + 3D	10.7	−1.4	1.5	24	94.3
Proposed	40	89	20	125	89.25

## Data Availability

The data that support the findings of this study are available on request from the corresponding author.
